# Research Progress of Ferroptosis: A Bibliometrics and Visual Analysis Study

**DOI:** 10.1155/2021/2178281

**Published:** 2021-08-06

**Authors:** Jian Xiong, Wenchuan Qi, Jiacheng Liu, Zhenqing Zhang, Ziwen Wang, Jinku Bao, Chuanfang Wu, Fanrong Liang

**Affiliations:** ^1^Chengdu University of Traditional Chinese Medicine, Chengdu 610075, China; ^2^Guangxi University of Traditional Chinese Medicine, Nanning 530001, China; ^3^Key Laboratory of Bio-Resource and Eco-Environment of Ministry of Education, College of Life Sciences, Sichuan University, Chengdu 610041, China

## Abstract

**Background:**

Ferroptosis is a type of cell death with major topic of debate under current research and plays an important role in disease regulation.

**Objective:**

In this study, the literature management software Bibexcel and knowledge graph tool VOSviewer were used to summarize and analyze the international research trends and hotspots about ferroptosis in recent years, which highlight the disease mechanism, diagnosis, and treatment related to ferroptosis. *Material/Methods*. The core collection database of Web of Science was used for retrieving ferroptosis research literature. The information such as the amount of text, the country, the period, the institution, the fund, and the keywords was extracted by the bibliometric tool Bibexcel. The cooccurrence and clustering function of VOSviewer were used to analyze the high-frequency keywords and the cooperative network of the author, institution, and country.

**Results:**

The research of ferroptosis started late and was formally proposed in 2012. It has developed rapidly and presented an “exponential” growth trend. China, the United States, Germany, Japan, and France are the main national forces of ferroptosis research development. The United States and China have a relatively high degree of support and attention to ferroptosis. Exploring oxidative stress, inducers/inhibitors, synergistic antitumor effect, relationships with other cell death types, GSH/GPX4 and iron metabolism imbalance related mechanisms of ferroptosis, and ferroptosis in the nervous system disease, ischemia-reperfusion injury, tumor, inflammation, and age-related diseases are the hot research directions.

**Conclusion:**

Ferroptosis has been a research hotspot in the field of biomedicine in recent years and has attracted the attention of scholars all over the world. The occurrence mechanism of ferroptosis and its application in neurological diseases, ischemia and reperfusion injury, tumors, inflammation, and aging are the hot directions of current research. In the future, ferroptosis can be appropriately considered for strengthening new approaches, new diseases, new inductors, new inhibitors, clinical transformation, and traditional medicine research.

## 1. Introduction

Ferroptosis is an iron ion-related metabolic abnormality with the main feature of lipid peroxidation programmed cell death which has caused extensive attention in recent years. Its gene expression, reaction molecules, biochemical characteristics, and influence morphology are different from other known cell death types: apoptosis, autophagy, necrosis, and pyroptosis. The related mechanisms of ferroptosis such as iron metabolism imbalance, oxidative stress, abnormal glutamate metabolism, and lipid metabolism are involved in the occurrence and development of many diseases and have common mechanisms with the pathological changes of many diseases. These original and important discoveries provide new potential targets for the prevention and control of ferroptosis related diseases. Current evidence shows that ferroptosis plays an important role in ischemia-reperfusion injury, tumor disease, renal failure, circulatory system disease, and nervous system disease [1]. Therefore, it is of positive significance to summarize the existing research results of ferroptosis, discuss the research trends and frontier hotspots of ferroptosis, and reveal the new detailed molecular targets and mechanisms of ferroptosis in depth.

At present, many research summaries and analyses are often confined to literature reading combined with personal experience, lacking a general overview and overall grasp. In this study, literature management software Bibexcel and knowledge map tool VOSviewer were used to conduct bibliometric and visual analysis of ferroptosis. Through the analysis of literature keywords, authors, countries, institutions, funds, and cocitations in the field of ferroptosis research, it explores its research background, research status, research hotspots, and dynamic trends. It hopes to provide references and suggestions for the research on the pathogenesis and clinical application of ferroptosis in the future.

## 2. Materials and Statistical Analysis

### 2.1. The Data Source

The literature in this study is mainly from the Web of Science core collection database, Science Citation Index Expanded. The timeline is limited to 2020 from the beginning of the construction of the database. The types of literatures were restricted to ARTICLE and REVIEW, and two researchers independently searched and screened the literatures with TS = (“Ferroptosis” OR “Iron Death”), regardless of language. The search date was December 17, 2020. A total of 1,363 effective literatures were obtained.

### 2.2. Statistics and Analysis

After selecting the valid documents related to the research, they were downloaded and saved in plain text format. Bibexcel was used to extract the number of papers, year, journal, country, fund, and keywords from the effective bibliography, and the software was used to calculate the H-index of the corresponding author. The H-index indicates that the author's H paper has been cited at least H times at most. The H-index can accurately evaluate and reflect the academic achievement and level of researchers, so as to discuss and compare the contributions of researchers to the field [2]. The research results show that the higher the H-index value, the higher its quantity, quality, and academic influence. Frequency statistics and keyword analysis of VOSviewer 1.6.15 and Pajek5.13 were used to perform biclustering analysis of high-frequency keywords, and VOSviewer software network analysis and density analysis modules for visual map analysis were used so as to objectively reflect research hotspots. The author's collaboration network, institutional collaboration network, and country-regional collaboration network visualized collaborative analysis were all realized through VOSviewer [3, 4], which provides guidance and reference for scholars to understand the current situation of cooperation in the research field and carry out extensive scientific research cooperation. Data entry, analysis, and verification were independently completed by two researchers. The rest of the chart-making and analysis were done in Excel 2013.

## 3. Results

### 3.1. Basic Features of the Literature

#### 3.1.1. Distribution of Publication Output

From 2012 to 2020, A total of 1363 articles related to the ferroptosis field can be collected. The number of publications in the field of ferroptosis is increasing, overall showing the “exponential” rapid growth. It shows that ferroptosis research is in its development process of “growing period” with a great potential to grow. The earliest research was carried out in 2012. After 2018, the number of published articles was more than 100, and the number of published articles was the highest in 2020. This indicates that the research of ferroptosis has been the focus of scholars' attention in recent years and is a hot research direction of future medical research (Figure 1).

#### 3.1.2. Distribution of Country

Through Bibexcel software, a scientific metrological analysis is made of the national characteristics of ferroptosis research. The results show that more than 100 papers were published in four countries, accounting for 96.99% of the total number of papers published. The top 5 countries are China, the United States, Germany, Japan, and France (Table 1), indicating that these 5 countries are the core strength of international ferroptosis research field. In addition, the number distribution map of the world presents that Eastern Asia, North America, Europe, and Oceania are the core region for ferroptosis research, which is basically in line with the world's regional economic, social, and cultural level of spatial distribution pattern. China located in the Eastern Asia region is the rapid development country of ferroptosis research, but the average cited frequency and H-index are on the low side (Figure 2).

#### 3.1.3. Distribution of Academic Journals

The journals of ferroptosis were analyzed, the number of journals was counted, as well as citations and influencing factors, and the number of articles published by the top 10 journals accounted for 18.78% of the total number of articles published. Among them, more than 30 papers have been published in “Cell Death and Disease,” “Biochemical and Biophysical Research Communications,” and “Free Radical Biology and Medicine.” Combining the influencing factors and citations of major journals, it can be found that “Cell Death & Disease,” “Free Radical Biology and Medicine,” “Redox Biology,” “Cell Death and Differentiation,” and “Oxidative Medicine and Cellular Longevity” are also high-impact journals with an impact factor over 5 (Table 2). To a certain extent, such journals can be regarded as the main position and representative of ferroptosis. Well-known journals about cytology, biomolecular science, comprehensive medicine, and oncology have shown greater interest and tendency in the research of ferroptosis, reflecting the comprehensiveness and intersectionality of the research.

#### 3.1.4. Distribution of Funding Institutions

The funded projects of the thesis results often reflect the attention rate of the country and institutions to the research field and also represent the development trend of the corresponding research, the existing research resources, and the research level of related fields [5]. In these 1363 articles, a total of 5095 funds were found (Table 3). Five of the top 10 publications funded by projects in the United States are leading. They are National Institutes of Health (NIH), USA, United States Department of Health Human Services, NIH National Cancer Institute (NCI), NIH National Institute of General Medical Sciences (NIGMS), and NIH National Institute of Neurological Disorders Stroke (NINDS). In addition, the number of published papers funded by the National Natural Science Foundation of China is 427, ranking first (Figure 3). Although in essence academic output level and academic output quantity are not necessarily related to funding projects, it can be found that the support and attention from the United States and China to the field of ferroptosis research are still relatively leading.

#### 3.1.5. H-Index of Main Authors

Before the development and application of the Hirsch index, various indicators for evaluating the personal influence of researchers had their own advantages. Compared with other indicators, the H-index can organically combine the researcher's output and influence through algorithm technology, thus comprehensively considering the “quality” and “quantity” of academic achievements [6].  Table 4 lists the H-index value and the total number of citations of the top 15 authors whose H-index was more than 10. Judging from the essential significance of Hirsch index, 7 of the authors with an H-index more than 10 are from the United States, accounting for 46.7%, mainly from Columbia University and the University of Pittsburgh. This shows that these universities and research institutions have scientific research resources in the field of ferroptosis with the leading level in the world. At the same time, three Chinese authors, Tang Deli, Wang Hao, and Wang Xu, whose H-index exceeds 10, show that they play an indispensable role in the field of ferroptosis and have a certain influence.

### 3.2. Visual Analysis

#### 3.2.1. Analysis of the Author Partnership Network

A visual analysis of the collaborative network of authors who published more than 7 papers is shown in Figure 4. The size of the dots indicates the academic influence and cooperation degree of authors; the width of the line between the dots indicates the strength of the cooperative relationship between corresponding authors; and the color indicates the subcluster network to which the authors belong. Author's network of cooperative relations of ferroptosis presents the characteristics of “overall dispersion and multicenter and regional concentration.” “Tang DL”-“Kang R,” “Stockwell BR,” “Conrad M,” and “Angeli JPF” formed a larger net cooperation subgroup and branch outward radiation. Exploring the author collaboration network relationship can fully show the research achievements communication situation in the field.

#### 3.2.2. Analysis of Cooperation Network Relationship about Institutions

The analysis of the cooperative network of institutions that have published more than 10 papers is shown in Figure 5. The size of the dots indicates the academic influence and cooperation degree of the institutions; the width of the lines between the dots indicates the strength of the cooperative relationship between the corresponding institutions; and the color represents the subcluster network to which the institutions belong. There were roughly 6 major cooperative subclusters. In cluster 4, the number and the quantitative index of “Univ Pittsburgh” ranked first. According to the literature, the University of Pittsburgh has cooperated with 11 organizations such as “Guangzhoumeduniv” and “Centsuniv.” The University of Pittsburgh researchers have succeeded in deciphering the ferroptosis trigger signals language in cell, in 2020. “Univ Pittsburgh” associated with “Jinan University” found iPLA2*β* is an important regulatory protein for ferroptosis. The accumulation of lipid peroxides caused by loss of activity is closely related to the occurrence of Parkinson's disease. Inhibition of ferroptosis is expected to be a new strategy for the treatment of Parkinson's disease [7]. In cluster 1, “Chinese Acad Sci”-“Zhejiang Univ”-“Shanghai Jiao Tong Univ” as representatives of Chinese university and research institutions accounted for 27.1% of the total. Professor H. D. Wang from Zhejiang University and others from Zhengzhou University have discovered a drug for rheumatoid arthritis known as Auranofin; it can significantly activate Hepcidin and effectively reduce the iron overload burden. Furthermore, the researchers found that the molecular mechanism for this phenomenon is to reduce iron overload by activating the NF-*κ*B/IL-6/JAK-STAT signaling pathway [8]. In 2020, together with the Chinese Academy of Medical Sciences and others, Professor H. D. Wang clarified the effect and molecular regulation mechanism of ferritin inhibiting the occurrence of cardiomyopathy by regulating ferroptosis. It was first revealed in vivo that membrane protein SLC7A11 can effectively reverse cardiomyopathy caused by ferritin deficiency by blocking ferroptosis in cardiomyocytes, which is expected to become a new target for the prevention and treatment of heart diseases [9]. University of Science and Technology of China (USTC) and others jointly found that monodispersed amorphous Fe carbonate containing nanodrug assembly (calcium carbonate based Fe2+ -adriamycin complex, ACC@DOX.Fe2+ -CASI-PAMAM-FA/MPEG) can synergically induce ferroptosis and apoptosis of tumor cells [10]. In cluster 2, “Columbia Univ”-“Stanford Univ”-“Harvard Med Sch” asrepresentatives of university and research institutions accounted for 21.4% of the total. In 2017, Columbia University in the United States, as the origin and core institution of ferroptosis research, invited researchers from 27 institutions around the world to publish a programmatic guide on ferroptosis research, systematically expounding the mechanism of ferroptosis and its relationship with human diseases [11]. In cluster 3, “Jilin Univ”-“Univ Melbourne”-“Shandong Univ” as representatives of universities and research institutions in China and Australia accounted for 18.5% of the total. Sun et al. from Jilin University published their important research results, discussing how to regulate ferroptosis and lipid metabolism abnormality through overexpression and knockdown of perilipin2, a potential predictive biomarker in gastric cancer [12]. In cluster 5, “Helmholtz Zentrum Munchen”-“Johannes Gutenberg Univ Mainz”-“Univ Wurzburg” as representatives of German research institution groups accounted for 11.4% of the total. “Targeting Ferroptosis: New Hope for As-Yet-Incurable Diseases” was published in Trends in Molecular Medicine by Marcus Conrad, Svenja M.Lorenz, and Bettina Proneth form the German Institute for Metabolism and Cell Death in October 2020. This paper argues that because ferroptosis pathway provides a variety of drug-addable nodes, it is expected that the preclinical and clinical development of ferroptosis modulators will bring about unprecedented opportunities for treating uncured diseases [13]. In cluster 6, German research group with the core of “Univ Ghent” accounted for 5.7% of the total.

#### 3.2.3. Analysis of the Network of Country Cooperation

An analysis of the country cooperation relationship with 5 or more papers published is shown in Figures 6 and 7. The size of the dot indicates the academic influence and degree of cooperation of a country; the width of the line between the dots indicates the strength of the cooperation relationship between the corresponding countries; the color indicates the subcluster network to which they belong. The results of the study show that the United States, China, and Germany have close cooperative relations, and the overall performance of international cooperation is good. It can be seen from the network map of China's scientific research cooperation that China maintains scientific research cooperation with many countries such as the United States, Germany, France, Sweden, Japan, Australia, and Russia. Strengthening international cooperation is an important factor in promoting the output, dissemination, and commercialization of high-quality research results. While integrating into the internationalization process of frequencies and strengthening cooperation between countries, China should also focus on its own independent innovation and improvement of original results in order to enhance its influence and voice in this field.

#### 3.2.4. Cooccurrence and Cluster Analysis of Keywords

Summarizing the themes of keywords and analyzing keywords can help understand the research hotspots and trends in this field. In this study, VOSviewer software was used to extract the cooccurrence frequencies of more than 8. Cluster analysis with 64 keywords was performed. The 53 keywords were divided into 6 categories, combined with the meaning and logical analysis of the research subject words between the words, as shown in Figure 8: (1) oxidative stress response of ferroptosis and its application in stroke, Alzheimer's disease, and breast cancer (red): iron drop, active oxygen, iron overload, antioxidants, iron, mitochondria, stroke, Alzheimer's disease, oxidative stress, induced labor, nrf2, and breast cancer; (2) the inducer/inhibitor of ferroptosis response and its role in cerebral hemorrhage and diseases of aging (yellow): erastin, ferrostatin-1, cerebral hemorrhage, Fenton reaction, and aging; (3) ferroptosis mechanism involved in antitumor research (sky blue): sorafenib and pancreatic cancer; (4) relationship between ferroptosis and other cell death types, where ferroptosis is involved in inflammation and ischemia-reperfusion (dark blue): autophagy, cell death, pyroptosis, necroptosis, and apoptosis; (5) ferroptosis glutathione and peroxidase-4 systems and antimelanoma and glioma studies (purple): melanoma, glutathione, glioma, and GPX4; (6) correlation between iron metabolism imbalance and tumor microenvironment and antitumor genes (green): cancer stem cell, iron metabolism, tumor microenvironment, and p53.

The density view of the VOSviewer software was used to perform cooccurrence analysis on keywords (Figure 9). The frequency of keyword occurrences is related to the image density. The higher the frequency, the darker the color and the higher the density. At the same time, with larger gray value of the color, it also represents the bias of the research hotspot in this field. The keywords in the middle area of the figure are divided into five parts according to their location distribution, similar to the result of keyword clustering analysis. The first part is in the center of the view. Keywords were the following: iron drop disease, reactive oxygen species, iron overload, cancer, p53, and metabolism; the darkest part indicates that it is an international research hotspot in this field. Among them, ferroptosis has a large hotspot distribution area and is a high-frequency keyword. The oxidative stress response, iron metabolism, tumor, and tumor suppressor genes of ferroptosis occupy the core research position. The second part is located at the bottom left of the first part. The keywords were iron, Alzheimer's disease, oxidative stress, mitochondria, and stroke, focusing on the application of ferroptosis in stroke, Alzheimer's disease, and other neurological diseases. The third part is mainly located at the bottom right of the first part. Taking necrosis, scorch, apoptosis, and autophagy as keywords, this part focuses on the relationship between ferroptosis and other types of cell death. The fourth part is mainly located at the upper right of the first part. The keywords were glutathione, glioma, and GPX4, mainly related to glutathione and its peroxidase 4. The fifth part is mainly located on the upper part of the first part. Keywords were iron metabolism and tumor microenvironment, focusing on the research about abnormal iron metabolism, tumor microenvironment, and tumor stem cells.

## 4. Discussions

### 4.1. International Ferroptosis Research Development Trend

In this study, bibliometrics and visual analysis were used to make a macroscopic description and retrospective analysis of the research literature on ferroptosis, presenting research trends, hotspots, topics, major researchers, major research institutions, important research journals, and funding in this field. In recent years, a large number of literatures about ferroptosis have been published, showing an “exponential” rapid growth trend, which is the focus of international medical research and a hot research direction. By combining the historical axle of landmark research achievements on ferroptosis (Figure 10) and the number of published articles (Figure 1), the research on ferroptosis started late, officially in 2012. Dixons et al. [14] formally proposed the concept and characteristics of ferroptosis. In 2014, Yang et al. [1] found that GPX4 can regulate the death of eosinophilic cancer cells through the ferroptosis pathway. In 2016, ferroptosis inducers inhibited GPX4 by covalently targeting the active site selenocysteine, leading to accumulation of PUFA hydroperoxides [15]. In 2017, Doll et al. [16] found that ACSL4 inhibition is an important mechanism to improve the occurrence of ferroptosis. In 2018, Ingold et al. [17] found that GPX4 was selenium-dependent in preventing ferroptosis caused by hydrogen peroxide. In 2019, FSP1 is a key component of a nonmitochondrial coantioxidant system that acts in parallel with the GPX4 pathway based on glutathione [18]. In 2020, Zou et al. [19] revealed the role of peroxisomal-ether-phospholipid axis in the development of susceptibility and avoidance of ferroptosis and emphasized that PUFA-EPL is a unique functional lipid class, which is dynamically regulated in the process of cell state transition and provides multiple regulatory nodes for therapeutic intervention of disease. Zhou and Jinku [20] established a database of manually collected and managed ferroptosis-related markers and regulators and ferroptosis-related diseases.

### 4.2. Ferroptosis Research of High-Influence Scholar-Institution-Country and Cooperative Relationship

Stockwell BR (Columbia University), Conrad M (Helmholtz Zentrum Munchen), Linkermann A (Dresden University of Technology), Tang DL (Guangzhou Medical University), and Kang R (University of Pittsburgh) are influential in the field of ferroptosis. The cooperation between authors has increased, including interorganizational cooperation and international cooperation. Author-institution-country has a certain correlation in the number of papers published. China, the United States, Germany, Japan, and France are the countries with the biggest numbers of publications. There are many highly productive scholars in China, the United States, and Germany, and the team of them cooperates closely with the international community. A large-scale research team has initially formed, and each research direction has its own characteristics. However, it is also necessary to strengthen interagency and interregional cooperation and carry out high-quality academic exchanges and cooperation.

### 4.3. Ferroptosis Research Fund Support and Main Journal Position

The scientific research results of funded projects often reflect the attention rate of the country and institutions. The number of papers in the journals about the research field can reflect the interests of the journals and provide a reference to the paper publication and hot follow-up research information. The National Natural Science Foundation of China, National Institutes of Health (NIH), U.S. Department of Public Services, National Institutes of Health National Cancer Institute (NCI), and National Institutes of Health National Institute of General Medical Sciences (NIGMS) are the main fund project institutes in supporting ferroptosis research with a positive significance. The journals with the highest output are “Cell Death and Disease,” “Biochemical and Biophysical Research Communications,” “Free Radical Biology and Medicine,” “Redox Biology,” and “International Journal of Molecular Science.” To a certain extent, this reflects the status of major journals in the study of ferroptosis. However, due to the limitations of space and review requirements, the publication of research results from top international journals cannot be ignored. Secondly, the study of ferroptosis is a multidisciplinary research topic, which can be further explored from the perspective of diseases in various disciplines.

### 4.4. Analysis of Ferroptosis Research Hotspot Trend

The visualization analysis of keyword clustering found that 53 keywords were clustered into 6 topic directions. Oxidative stress, inducers/inhibitors, synergistic antitumor effect, relationships with other cell death types, glutathione peroxidase, GPX4, and iron metabolism imbalance related mechanisms of ferroptosis were discussed. The application of ferroptosis in nervous system diseases, ischemia-reperfusion injury, tumor, inflammation, and aging related diseases is a hot research direction (Figure 8; Table 5).

#### 4.4.1. Oxidative Stress Response of Ferroptosis and Its Application in Stroke, Alzheimer's Disease, and Breast Cancer

Cluster 1 (red) of keywords focuses on ferroptosis oxidative stress and its application in stroke, Alzheimer's disease, and breast cancer. Oxidative stress is a reaction process in which reactive oxygen species generated during the aerobic metabolism of the body accumulate excessively in cells, leading to cell damage and death. Its essence is the imbalance between the body's [21] antioxidant defense and the production of reactive oxygen species. The mechanism of ferroptosis is due to the damage of the glutathione- (GSH-) dependent lipid peroxide repair system, which leads to the accumulation of reactive oxygen species in lipids [11, 14]. Mitochondrial electron transport chain complex I inhibitor DPI can inhibit oxidative stress response [22], and mitochondrial complex III inhibitor antimycin A can inhibit erastin-induced ferroptosis [14, 23], indicating that both ferroptosis and oxidative stress pathways rely on mechanisms for GSH reduction and related antioxidant system damage. A large number of studies have shown that ferroptosis is an important potential target for stroke prevention and treatment. Inhibition of ferroptosis response can reduce stroke injury [24–28], and its mechanism is related to excitement related to iron overload [28], ACSL4 protein [29], 12/15-LOX expression [30], XCT expression [31], and increased sexual toxicity. Abnormal iron metabolism plays an important role in the occurrence and development of Alzheimer's disease. Patients with Alzheimer's disease have obvious iron deposits in the cerebral cortex and hippocampus, which corresponds to the distribution of A*β* plaques [32, 33]. Elevated iron content in the brain can aggravate the disease, and A*β* accumulation [33] and iron chelating agents can reduce the level of iron in the brain and relieve symptoms [34]. Cys deletion in triple-negative breast cancer (TNBC) cells can induce ferroptosis, and DFO and Tistatin-1 can block the corresponding cell death [35]. Ferroptosis may also mediate the synergistic anti-breast-cancer effect of cyclamine and lapatinib [36].

#### 4.4.2. The Inducer/Inhibitor of Ferroptosis Response and Its Role in Cerebral Hemorrhage and Diseases of Aging

Cluster 2 of keywords (yellow) mainly focuses on the inducer/inhibitor of ferroptosis response and its role in cerebral hemorrhage and diseases of aging. Erastin is a classic inducer of ferroptosis reaction, which can inhibit System XC- activity and affect glutathione (GSH) synthesis, combined with VDAC2/3 inducing mitochondrial dysfunction [14, 22, 37]. Ferrostatin1 classical inhibitor of ferroptosis reaction eliminates lipid reactive oxygen species (ROS), inhibits lipid peroxidation, regulates the expression of oxidization-related proteins, and reduces unstable iron in cells [14, 38–43]. Intracerebral hemorrhage injury also has the phenomenon of neuronal ferroptosis [44]. Intracerebral hemorrhage injury can be alleviated by the administration of ferroptosis inhibitors, the mechanism of which is mainly related to iron overload [45], decreased expression of glutathione peroxidase 4 [46], and increased activity of arachidonic acid-dependent lipoxygenase-5 (ALOX5) [47]. Aging can cause excessive accumulation of iron ions in cells, damage DNA, and inhibit the ability to repair DNA damage, while incomplete DNA loss accelerates cellular neurodegeneration and aging of the body [48, 49]. The mechanism may be that iron ions take up the binding site of p53 protein, thus weakening p53 to repair DNA damage [49].

#### 4.4.3. Ferroptosis Mechanism Involved in Antitumor Research

Cluster 3 of keywords (sky blue) mainly focuses on ferroptosis mechanism involved in antitumor research. Sorafenib is a clinical multitargeted antitumor drug and also an important inducer of ferroptosis. Deferriamine can block the oxidative stress response induced by sorafenib in HCC HUH7 cells, suggesting that the antitumor targeting effect of sorafenib may be mediated through the ferroptosis pathway [50]. Sorafenib can induce the expression of metallothionein-1G (MT-1G) gene in liver cancer cells, thereby inhibiting ferroptosis and promoting drug resistance [51, 52]. Studies have shown that inhibition of p62-KEAP1-Nrf2 antioxidant signaling pathway can significantly enhance the anti-HCC activity of erastin and sorafenib, indicating that the induction of ferroptosis can promote the anti-HCC targeted sensitization of erastin and sorafenib [53]. Sorafenib and low-dose PDT have a synergistic effect in inhibiting tumor progression, and the mechanism may be to reshape tumor immune microenvironment by inducing T cell-dependent local and systemic antitumor immune response [54].

#### 4.4.4. Relationship between Ferroptosis and Other Cell Death Types: Ferroptosis Is Involved in Inflammation and Ischemia Reperfusion

Cluster 4 of keywords (dark blue) mainly focuses on the relationship between ferroptosis and other cell death types. Ferroptosis is involved in inflammation and ischemia-reperfusion. The morphology of ferroptosis is different from those of apoptosis, necrosis, and autophagy. Ferroptosis is mainly manifested as mitochondrial atrophy, cristae disappearance, increased membrane density, and outer membrane rupture [14]. In the past, inhibitors widely used for apoptosis, necrosis, or autophagy could not prevent ferroptosis. However, there is a certain correlation between ferroptosis and other types of cell death. Under certain conditions, cell apoptosis can be transformed into ferroptosis, which also can promote the sensitivity of cells to apoptosis. The tumor suppressor gene p53 can not only fight tumors through cell cycle arrest and apoptosis but also induce ferroptosis reactions in tumor cells under certain conditions. Studies have shown that autophagy activation can degrade ferritin, leading to ferroptosis in tumor cells [55]. Ferroptosis may be the process of autophagy death, which is induced by autophagy [56]. Ferroptosis and programmed necrosis are complementary forms of cell death. When the programmed necrosis pathway is weakened, ferroptosis pathway becomes more sensitive [57]. Ferroptosis is often related to the inflammatory immune process, and the two are closely related. In acute kidney injury (AKI) model and tamoxifen-induced systemic GPX4 deletion knockout mice, it is shown that inflammation is associated with ferroptosis of the kidney [58]. The significant activation of macrophages is observed through the development of ferroptosis tissues involved in the inflammatory response [59]. The occurrence of pancreatic cancer is related to iron metabolism and lipid peroxidation. The possible mechanism of antitumor action of Ruscogenin is to regulate transferrin to increase intracellular Fe ion concentration, inducing ferroptosis [60]. The activation of the Atg5/Atg7-NCoA4 axis in pancreas cancer PANC-1 cells can degrade ferritin, inhibit the expression of the heavy chain of ferroprotein, and induce ferroptosis [61]. In the study of pancreatic cancer PANC-1 cells, the antioncogene p53 may exert a tumor suppressor effect through the ferroptosis mediated by the SAT1-ALOX15 axis [62].

#### 4.4.5. Ferroptosis Glutathione and Peroxidase 4 Systems, Antimelanoma, and Glioma Studies

Cluster 5 of keywords (purple) mainly focuses on ferroptosis glutathione and peroxidase 4 system and antimelanoma and glioma research. Cystine/glutamate antiporter system XC- is exchanged between intracellular cystine and glutamate in a 1 : 1 ratio, and extracellular glutamate accumulation is an important regulator of ferroptosis [56]. Glutathione (GSH) is the main substrate of glutathione peroxidase 4 (GPX4), a key regulator of death [63]. Inhibition of GPX4 can induce a large number of lipid peroxides to aggregate in cells and form a marker reaction of ferroptosis [64]. Melanoma is a kind of skin tumor with high malignant degree, and miR-137 can mediate the glutamine transporter SLC1A5 to regulate the occurrence of ferroptosis in melanoma cells [65]. Erastin, a classic inducer of ferroptosis, can significantly enhance the killing ability of vemurafenib against M229R and M238R melanoma cells [66]. Activation of ferroptosis in glioblastoma stem cells increases the sensitivity of tumor cells to temozolomide, opening a new pathway for glioblastoma therapy [67–69].

#### 4.4.6. Correlation between Iron Metabolism Imbalance and Tumor Microenvironment and Antitumor Genes

Cluster 6 of keywords (green) mainly focuses on the correlation between iron metabolism imbalance and tumor microenvironment and antitumor genes. Iron is an important factor in the accumulation of lipid peroxides in ferroptosis. Iron metabolism imbalance and ferritin autophagy are important regulatory targets for ferroptosis. Iron responsive element binding protein 2 (IREB2) can mediate transferrin and transferrin receptor iron import cells to induce ferroptosis, and silencing the IREB2 gene can inhibit ferroptosis [56]. This process is affected by IREB2 [14]. Autophagy can also affect the iron metabolism pathway and regulate the ferroptosis response [70, 71]. p53 is an important tumor suppressor molecule, which can induce the occurrence of ferroptosis and mediate its antitumor effect through the sensitivity of cells to ferroptosis. p53 can inhibit the SLC7A11-induced ferroptosis response through a transcription-dependent pathway and play a role in suppressing tumors [72, 73]. It is found that p53 can delay ferroptosis, and erastin does not significantly stimulate the ferroptosis of p53 in colorectal cancer (CRC). Inhibition or knockout of p53 can restore the ferroptosis response caused by erastin [74], indicating that p53 plays a complicated role in the death mechanism of ferroptosis cells, and further research is needed.

## 5. Conclusion

This article studies the English literature of ferroptosis published in the Web of Science core collection database. The earliest article to clarify the concept of ferroptosis was published in 2012, and the number of articles presents an exponential growth trend, indicating that ferroptosis research started late and has been a hot research spot in the field of biomedical science in recent years. It has attracted wide attention from scholars all over the world. The occurrence mechanism of ferroptosis is the hot directions of current research. In terms of disease carrier selection, stroke, Alzheimer's disease, cerebral hemorrhage, ischemia and reperfusion, inflammation, aging, breast cancer, liver cancer, melanoma, and glioma are the key subjects of the current ferroptosis mechanism-related disease research. Secondly, is there a new way in the study of the action mechanism of ferroptosis? Can new inductors and inhibitors of ferroptosis be screened? What are the complete mechanism and pathway for ferroptosis involved in anti-inflammatory and antitumor activation of the immune system? Can the research results of antitumor mechanism based on ferroptosis be better applied and transformed into clinical front-line? Discuss the relationship between traditional medicine and ferroptosis. These issues still need extensive and thorough research.

## Figures and Tables

**Figure 1:** Number of annual publications.

**Figure 2:** Distribution of countries with more than 10 publications.

**Figure 3:** Top 10 fund organizations and number of publications.

**Figure 4:** Cooperative network of individual authors.

**Figure 5:** Institutional cooperation network.

**Figure 6:** National cooperation network.

**Figure 7:** Chinese network of cooperation with other countries.

**Figure 8:** Keyword clustering visualization.

**Figure 9:** Density map of keywords.

**Figure 10:** Historical axis of landmark achievements in ferroptosis research development.

**Table 1:** Country distribution (top 10).

Rank	Country (region)	Freq.	Total citation frequency	The average cited frequency	H-index
1	China	620	10828	17.46	73
2	USA	434	22377	51.56	48
3	Germany	161	9366	58.17	45
4	Japan	107	4264	39.85	25
5	France	62	2982	48.10	25
6	Australia	51	3010	59.02	22
7	UK	50	3752	75.04	20
8	Canada	46	2092	45.48	18
9	Italy	44	1539	34.98	17
10	Russia	35	1640	46.86	15

**Table 2:** The characteristics of main academic journals publications about ferroptosis (top 10).

Rank	Journals	Publications	Total citation frequency	The average cited frequency	Impact factor
1	Cell Death and Disease	45	588	13.07	6.486
2	Biochemical and Biophysical Research Communications	36	904	25.11	2.75
3	Free Radical Biology and Medicine	31	1112	35.87	6.457
4	Redox Biology	27	740	27.41	9.789
5	International Journal of Molecular Sciences	25	200	8.00	4.653
6	Cell Death and Differentiation	22	1999	90.86	9.597
7	Oxidative Medicine and Cellular Longevity	20	193	9.65	5.608
8	Scientific Reports	18	237	13.17	4.576
9	Frontiers in Neuroscience	16	261	16.31	2.649
10	Cancers	16	56	3.50	6.433

**Table 3:** Funds distribution (top 10).

Rank	Fund subvented organizations	Number of literatures (articles)
1	National Natural Science Foundation of China (NSFC)	427
2	National Institutes of Health (NIH), USA	307
3	United States Department of Health Human Services	307
4	NIH National Cancer Institute (NCI)	160
5	NIH National Institute of General Medical Sciences (NIGMS)	93
6	German Research Foundation (DFG)	74
7	Ministry of Education, Culture, Sports, Science and Technology (MEXT), Japan	70
8	Japan Society for the Promotion of Science	61
9	Grants-in-Aid for Scientific Research (KAKENHI)	46
10	NIH National Institute of Neurological Disorders Stroke (NINDS)	40

**Table 4:** H-index of main authors (H-index more than 10).

Rank	Author	Country	Publications	Total citation frequency	The average cited frequency	H-index
1	Stockwell	USA	47	10054	213.91	33
2	Conrad	Germany	36	5059	140.53	26
3	Linkermann	Germany	28	4157	148.46	21
4	Tang	China	39	3525	90.38	20
5	Kang	USA	38	2418	63.63	20
6	Dixon	USA	25	5945	237.80	19
7	Angeli	Germany	21	3164	150.67	16
8	Kagan	USA	25	2628	105.12	14
9	Kroemer	France	14	1749	124.93	13
10	Bayir	USA	22	1913	86.95	12
11	Tyurina	USA	20	1770	88.50	12
12	Wang	China	21	623	29.67	11
13	Wang	China	18	370	20.56	11
14	Vandenabeele	Belgium	13	2790	214.62	11
15	Gu	USA	13	1154	88.77	11

**Table 5:** Keywords clustering table.

Clustering number	Color	Key keywords
Cluster 1	Red	Ferroptosis, reactive oxygen species, iron overload, antioxidant, iron, mitochondria, stroke, Alzheimer's disease, oxidative stress, oxytosis, nrf2, breast cancer
Cluster 2	Yellow	Erastin, ferrostatin-1, intracerebral hemorrhage, Fenton reaction, senescence
Cluster 3	Sky blue	Sorafenib, pancreatic cancer, ferritinophagy
Cluster 4	Dark blue	Autophagy, cell death, pyroptosis, necroptosis, apoptosis, inflammation, ischemia-reperfusion
Cluster 5	Purple	Melanoma, glutathione, glioma, GPX4
Cluster 6	Green	Cancer stem cell, iron metabolism, tumor microenvironment, p53, metabolism, cancer

## Data Availability

The data used to support the findings of this study are available from the corresponding author upon request.

## Additional Points

The limitation of visual analysis mainly lies in that some high-quality but low-impact factor literatures cannot analyze it, so as to provide more comprehensive suggestions for related research fields.
